# Association of Paraoxonase 1 Gene Polymorphisms with the Risk of Breast Fibroadenoma and Breast Cancer in the Females of Guangxi, China

**DOI:** 10.1155/2022/3642799

**Published:** 2022-03-08

**Authors:** Kun Chen, Xiaogang Wang, Dihang Li, Weiping Luo, Chuang Xue, Yong Kong

**Affiliations:** ^1^Department of Thyroid Gland and Breast Surgery, Guidong People's Hospital of Guangxi Zhuang Autonomous Region, Wuzhou 543001, Guangxi, China; ^2^Department of Medical Management, Guidong People's Hospital of Guangxi Zhuang Autonomous Region, Wuzhou 543001, Guangxi, China

## Abstract

Fibroadenoma of the breast is a common cause of a benign breast lump in premenopausal women. The consensus view is that women with fibroadenomas are not at significantly increased risk of developing breast cancer. The objective of this research was to explore the association of PON1 rs662 and rs705382 with the risk of breast fibroadenoma (BF) and breast cancer (BC) in the females of Guangxi in southern China. The PON1 rs662 and rs705382 single-nucleotide polymorphisms (SNPs) were genotyped by polymerase chain reaction-restriction fragment length polymorphism (PCR-RFLP) in 55 BF patients, 80 BC patients, and 98 healthy controls. Significant associations with FB and BC risks were observed for the rs662 SNP. Diagnosis is based on the combination of clinical examination, imaging, and nonsurgical tissue biopsy (the triple test) [21]. In haplotype analyses, the haplotype GA increases the risk and haploid GG decreases the risk in BF and BC. Our research indicated that the PON1 rs662 SNP might be a risk factor for BF and BC. The results of this research indicated that the locus of rs662 in PON1 is relevant to risk of developing BF and BC in the females of Guangxi. Further prospective studies are needed to support our conclusions.

## 1. Introduction

The single-nucleotide polymorphism (SNP) is the most frequent variation in human genome [1]. The human PON1 gene, encoded by the chromosome 7p21-22, contains 8 introns and 9 exons [2, 3]. PON1 is a kind of liver-induced sugar protease involved in anti-inflammatory and antioxidative mechanisms [4]. Cancer is often associated with oxidative stress, an outcome of which is a disruption in the balance between the systemic effects of toxic reactive species and the body's capacity to metabolize the excess free radicals and/or to repair the damage that they generate [5]. PON1 gene polymorphism has been proved to be related to malignant tumors [6, 7]. Breast cancer is the most frequently diagnosed cancer globally and is the leading cause of cancer-related deaths in women [8, 9]. It was proved that serum PON1 activity decreased in patients with breast cancer [10]. PON1 SNPs differences may affect the activities of PON1 enzyme and may lead to susceptibility of multiple diseases [11]. These associations deserve our discussion over the relation of PON1 SNPs and susceptibility to breast diseases. This research aims to explore the association of PON1 rs662 and rs705382 with the risk of breast fibroadenoma (BF) and breast cancer (BC) in females of Guangxi in southern China. In this research, we studied the association between SNPs of PON1 (rs662, rs705382) and genetic susceptibility of BF and BC in females of Guangxi. The results displayed that significant associations with BF and BC risk were observed for the rs662 SNP.

## 2. Materials and Methods

### 2.1. The Study Group

This study included 135 patients with breast diseases and 98 healthy controls. Patients were periodically recruited in Guidong People's Hospital of Guangxi Zhuang Autonomous Region, from January to December through October of 2017, including 55 BF patients and 80 FC patients. All diagnoses have pathological support. Members of the control group were randomly selected from the healthy females having body examination in the same hospital. Inclusion criteria: without other malignant tumors or other breast diseases, females from Guangxi. Signatures of informed consent were obtained from all objectives of the study. In addition, demographic characteristics and blood samples, including age, ethnicity, tobacco and alcohol use, and body mass index (BMI), were also collected by the interviewers. This study was approved by the ethics committee of Guidong People's Hospital of Guangxi Zhuang Autonomous Region.

### 2.2. DNA Extraction and Genotyping of PON1

The PON1 rs705382 and rs662 SNPs were genotyped by polymerase chain reaction-restriction fragment length polymorphism (PCR-RFLP). The PCR was carried out in 1.0 mL of each primer, 12.5 mL of Green PCR Master Mix (Shanghai Sangon Biotech Co., Ltd., Shanghai, China), 9.5 mL of sterilized deionized water, and 2.0 mL of template DNA per reaction. The forward and reverse primers used were rs662-F 5'-TATTGTTGCTGTGGGACCTGAG-3' and R 5'-CACGCTAAACCCAAATACATCTC-3' [12] and rs705382-F 5'-GAGAGGGAAAGTGGTCAGCT-3' and R 5'-GAAGTGTGAGTTTGGGCAGG-3'. The PCR reaction for rs662 included a 5-min preincubation step at 95°C, followed by 39 cycles of 45 seconds at 95°C, 45 seconds at 58°C, 45 seconds at 72°C, and then a final 10-min extension step at 72°C. For rs705382, it included a 5-min preincubation step at 95°C, followed by 24 cycles of 39 seconds at 95°C, 30 seconds at 56°C, 30 seconds at 72°C, and then a final 10-min extension step at 72°C.

After amplification, all products were separated on 3% agarose gel and subsequently stained with ethidium bromide to visualize the bands (Figures 1 and 2). To control the quality of the PCR reaction, a negative control was also performed in each genotyping assay. In addition, we entrusted Sangon Biotech to perform gene sequencing for 10% sample randomly chosen during the process for verification, which matches our results 100%.

## 3. Statistics Analysis

The Hardy-Weinberg equilibrium (HWE) was assessed by a goodness-of-fit chi-square test for genotypes in the control groups. For baseline data, 1-way analysis of variance (ANOVA) tests were used for the categorical variables, and student *t* tests were used for the continuous variables to compare the differences in demographic characteristics between patients and controls. Genotype and allele frequencies among different groups were compared using the chi-square test and Fisher exact test, when appropriate. Logistic regression analysis, adjusted for age, tobacco smoking, alcohol consumption, and BMI, was utilized to calculate the adjusted odds ratios (ORs) and 95% confidence intervals (CIs). The haplotype construction was performed using SHEsis software (http://analysis.bio-x.cn/myAnalysis.php). A probability level of less than 0.05 was judged as statistically significant. All statistical analyses were performed using SPSS, version 19.0 (SPSS Inc., Chicago, IL).

## 4. Result

### 4.1. Demographic Features

Demographic data of cases and controls are displayed in Table 1. Ages of BF group were significantly younger than the control group and the BC group (*P* < 0.001). BMI of this group was significantly lower than the other two groups (*P*=0.01). Breast cancer group was with significantly more history of smoking and drinking (*P* < 0.001). In comparison, the healthy control group was primarily without history of smoking and drinking, suggesting healthier way of living. Besides, significant differences exist in ethnic formation of three groups (*P*=0.002). In healthy controls, the observed genotype frequencies of rs662 and rs705382 were both in agreement with HWE (*P*=0.989, for rs662; *P*=0.849, for rs705382) Table 2.

### 4.2. Analysis of the Association between Gene Polymorphism and Risks of Developing BF and BC

Distribution of the rs662 genotype and allele was significant difference in three groups (*P* < 0.01). Adjusting age, ethnicity, history of smoking, history of drinking, and BMI with logic regression displayed significant correlation between the rs662 and the risks of developing BF and BC. Compared with GG genotype, AA genotype increased these risks more obviously; compared with allele G, allele A increased these risks more obviously. No obvious relevance were between the rs705382 and the risks of BF and BC (detailed in Table 3).

### 4.3. Haplotype Analysis of Associations between PON1 Polymorphism and BF and BC

We performed haplotype analysis for 4 haplotypes (CA, CG, GA, and GG). We found that haplotype GG is frequently seen in the control group and BC group. Haplotype CA ranked 1^st^ in BF group and 2^nd^ in control group and BC group (Table 4). The distribution of haplotype GA significantly increased risks of BC (OR = 3.239, 95% CI 1.705–6.152, *P* < 0.001). The distribution of haplotype GA significantly increased risks of BF (OR = 3.716, 95% CI 1.884–7.328, *P* < 0.001). The distribution of haplotype GG significantly decreased risks of BC (OR = 0.526, 95% CI 0.338–0.819, *P*=0.004). The distribution of haplotype GG significantly decreased risks of BF (OR = 0.389, 95% CI 0.230–0.658, *P* < 0.001).

## 5. Conclusion

PON1 is a kind of liver-induced sugar protease involved in the anti-inflammatory and antioxidative mechanism. In this research, we studied the association between SNPs of PON1 (rs662 and rs705382) and genetic susceptibility of BF and BC in females of Guangxi. The results displayed that significant associations with BF and BC risk were observed for the rs662 SNP. Haplotype analysis of the 2-candidate SNPs suggested haplotype GA is a risky factor of BF and BC. It was being reported that variation of rs662 and rs705382 locus in PON1 may have more influence on the activity of PON1 enzyme [13–15]. The SPNs rs662 locus influences hydrolysis capability of PON1 enzyme of lipid peroxide enzyme. Results of this research displayed significant relevance between rs662 locus of PON1 and incidence of BC and BF in females of Guangxi. The possible explanation may be that poor PON1 activity in female in Guangxi with homozygote AA carrying rs662 locus (geno-variation of homozygote) reacted poorly to emergency response and lipid peroxide response caused by cancer. As a result, the risks of developing these carcinomas are increased. The association of rs662 SNPs and genetic susceptibility of breast cancer were verified [16–19]. However, no research related to the association of rs705382 SNPs and breast diseases was found.

Analyzing multiple SNPs provides more meaningful results than only analyzing a single SNP [20]. The results of this research suggested that distribution of GA significantly increased (3.239 times) risks of BC and distribution of GA significantly increased (3.716 times) risks of BF.

Despite strong biological rationality and correlation of this research, there are several limitations need to be handled. Besides, the subject of this research is females in Guangxi, the relevant data may not suit other groups of females and need to be used cautiously. The results of this research indicated that the locus of rs662 in PON1 is relevant to risk of developing BF and BC in females of Guangxi. Further prospective studies are needed to support our conclusions.

## Figures and Tables

**Figure 1:** Electrophoretogram of rs662 locus enzyme-digested product. M lane for marker, lanes 1–12 were PCR enzyme-digested products of 12 specimens, the whole segment length was 99 bp, the lengths of enzyme-digested product segments were 3 bp and 36 bp, 6 for homozygote AA genotype, 1, 2, and 3 for homozygote GG genotype, and 4 and 5 for homozygote AG genotype.

**Figure 2:** Electrophoretogram of rs705382 locus enzyme-digested product. M lane for marker, lanes 1, 2, 3, 4, 5, and 6 were PCR enzyme-digested products of 6 specimens, the whole segment length was 577 bp, the lengths of enzyme-digested product segments were 368 bp and 208 bp, 1 and 2 for homozygote GG genotype, 3 and 4 for heterozygous CG, and 5 and 6 for homozygote CC genotype.

**Table 1:** Clinical and epidemiological data for the patient and control groups.

Parameters	Controls (*n* = 98, %)	BF (*n* = 55, %)	BC (*n* = 80, %)	*P* value
Age, *y*, mean SD	45.04 6.54	34.02 10.81	49.67 9.77	<0.001
BMI, mean SD	22.57 3.17	20.93 3.07	22.90 3.24	0.01
*Tobacco smoking*				
** **Yes	3 (3.1%)	4 (7.3%)	20 (25%)	<0.001
** **No	95 (96.9)	51 (92.7%)	60 (75%)	
*Alcohol drinking*				
** **Yes	7 (7.1%)	8 (14.5%)	19 (23.8%)	0.008
** **No	91 (92.9)	47 (85.5%)	61 (76.35%)	
*Ethnicity*				
** **Han	72 (73.5%)	49 (89.1%)	49 (61.3%)	0.002
** **Zhuang	23 (23.5%)	4 (7.3%)	30 (37.5%)	
** **Others	3 (3.1%)	2 (3.6%)	1 (1.3%)	

BMI = body mass index; BF = breast fibroadenoma; BC = breast cancer; SD = standard deviation.

**Table 2:** Genotype and allele frequencies of candidate SNPs in patients and control individuals.

Controls	BF	BC	*P* value
SNPs	*n* = 98 (%)	*n* = 55 (%)	*n* = 80 (%)
*rs662 genotypes*	HWE = 0.989			<0.001
** **GG	42 (42.9%)	22 (40.0%)	30 (37.5%)	
** **AA	11 (11.2%)	25 (45.5%)	26 (32.5%)	
** **GA	45 (45.9%)	8 (14.5%)	24 (30.0%)	
*rs662 alleles*				0.003
** **G	129 (65.8%)	52 (47.3%)	84 (52.5%)	
** **A	67 (34.2%)	58 (52.7%)	76 (47.5%)	
*rs705382 genotypes*	HWE = 0.849			0.583
** **CC	21 (21.4%)	14 (25.5%)	22 (27.5%)	
** **GG	24 (24.5%)	11 (20.0%)	23 (28.8%)	
** **CG	53 (54.1%)	30 (54.5%)	35 (43.8%)	
*rs705382 allele*				0.768
** **C	95 (48.5%)	58 (52.7%)	79 (49.4%)	
** **G	101 (51.5%)	52 (47.3%)	81 (50.6%)	

BF = breast fibroadenoma; BC = breast cancer.

**Table 3:** Genotype and allele frequencies of candidate SNPs in patients and control individuals.

Controls	BF			BC		
SNPs	*n* = 98 (%)	*n* = 55 (%)	OR (95% CI)	POR	*n* = 80 (%)	OR (95% CI)	POR
*rs662 genotypes*							
** **GG	42 (42.9%)	22 (40.0%)	1.00ref		30 (37.5%)	1.00ref	
** **AA	11 (11.2%)	25 (45.5%)	6.609 (2.077–21.022)	0.001	26 (32.5%)	3.862 (1.521–9.808)	0.004
** **GA	45 (45.9%)	8 (14.5%)	0.497 (0.161–1.532)	0.223	24 (30.0%)	0.569 (0.251–1.290)	0.177
** **GA + AA	56 (57.1%)	33 (60)	1.586 (0.659–3.818)	0.304	50 (62.5%)	1.193 (0.599–2.379)	0.615
*rs662 alleles*							
** **G	129 (65.8%)	52 (47.3%)	1.00ref		84 (52.5%)	1.00ref	
** **A	67 (34.2%)	58 (52.7%)	2.854 (1.529–5.328)	0.001	76 (47.5%)	1.878 (1.162–3.034)	0.01
*rs705382 genotypes*							
** **CC	21 (21.4%)	14 (25.5%)	1.00ref		22 (27.5%)	1.00ref	
** **GG	24 (24.5%)	11 (20.0%)	0.657 (0.187–2.312)	0.513	23 (28.8%)	0.925 (0.365–2.343)	0.869
** **CG	53 (54.1%)	30 (54.5%)	1.111 (0.387–3.195)	0.844	35 (43.8%)	0.579 (0.254–1.320)	0.194
** **CG + GG	77 (78.6%)	41 (74.5%)	0.949 (0.347–2.592)	0.919	58 (72.5%)	0.683 (0.317–1.471)	0.33
*rs705382 allele*							
** **C	95 (48.5%)	58 (52.7%)	1.00ref		79 (49.4%)	1.00ref	
** **G	101 (51.5%)	52 (47.3%)	0.826 (0.459–1.487)	0.524	81 (50.6%)	0.963 (0.603–1.538)	0.875

For rs662, codominant model: AG vs GG, GG vs GG, and dominant model: GA + AA. For rs705382, codominant model: CG vs CC, GG vs CC, and dominant model: CG + GG, adjusted for age, smoking, drinking, and BMI.

**Table 4:** Haplotype analysis of PON1 rs662 and rs705382 polymorphisms with the risk of BF and BC

			BF vs controls		BC vs controls	
Haplotype	Controls (n = 196, %)	BF (n = 110, %)	BC (n = 160, %)	OR (95% CI)	P_OR_	OR( 95% CI)	P_OR_
C a	26.30%	26.80%	25.80%	1.026 [0.605–1.740]	0.924	0.975 [0.606–1.569]	0.917
C G	22.20%	25.90%	23.60%	1.229 [0.714–2.117]	0.457	1.082 [0.658–1.779]	0.755
G a	7.90%	24.10%	21.70%	3.716 [1.884–7.328]	<0.001	3.239 [1.705–6.152]	<0.001
G G	43.70%	23.20%	28.90%	0.389 [0.230–0.658]	<0.001	0.526 [0.338–0.819]	0.004

BF = breast fibroadenoma; BC = breast cancer; CI = confidence interval; OR = odds ratio.

## Data Availability

The datasets used and/or analyzed during the current study are available from the corresponding author on reasonable request.
